RETRACTED

# Clinical Observation on the Effect of Systematic Nursing Intervention on Cognitive Function, Life Activity Ability, and Quality of Life of Senile Dementia Patients

**DOI:** 10.1155/2021/2839142

**Published:** 2021-10-12

**Authors:** Yuan Zheng, Xiaoyan Xu, Birong Zheng

**Affiliations:** ^1^Xi'an Health School, Xi'an, Shaanxi 710054, China; ^2^Department of General Practice, Jiangdong Branch of Zhuji People's Hospital, Zhuji, Zhejiang 311800, China

## Abstract

**Objective:**

To explore the influence of systematic nursing intervention on the life ability and quality of senile dementia patients.

**Methods:**

Total of 82 senile dementia patients who were admitted to our hospital from January 2018 to January 2020 were divided into two groups according to the random number table, and the nursing intervention was analyzed. 41 patients in the control group were given routine nursing care, and 41 patients in the observation group were given systematic nursing intervention. Patients were assessed cognitively using the Montreal Cognitive Assessment Scale (MoCA). The Barthel index and SF-36 were used to evaluate the patients' daily activity function and quality of life. A Symptom Checklist-90-Revised (SCL-90-R) was used to assess mental distress. The Social-Adaptive Function Rating Scale (SAFE) and Social Skills Inventory (SSC) were used to evaluate the patients' social interaction ability before and after nursing intervention. Nursing satisfaction was distributed to patients in the form of a self-prepared nursing satisfaction questionnaire for scoring.

**Results:**

After the nursing intervention, the MoCA scores of patients in the two groups were higher than those before the nursing intervention, and the scores in the observation group were higher than those in the control group (*P* < 0.05). After the nursing intervention, the Barthel index scores of patients in the two groups were higher than those before the nursing intervention, and the scores in the observation group were higher than those in the control group (*P* < 0.05). After the nursing intervention, the SF-36 scores of patients in the two groups were higher than those before the nursing intervention, and the scores in the observation group were higher than those in the control group (*P* < 0.05). After nursing intervention, the SCL-90-R scores of patients in the two groups were lower than those before nursing intervention, and the scores in the observation group were lower than those in the control group (*P* < 0.05). After the nursing intervention, the SAFE scores of patients in the two groups were lower than those before the nursing intervention, and the safe scores of the observation group were lower than those of the control group (*P* < 0.05). After the nursing intervention, the SSC scores of patients in the two groups were lower than those before the nursing intervention, and the scores in the observation group were lower than those in the control group (*P* < 0.05). After nursing intervention, the total satisfaction degree of the control group (80.49%) was lower than that of the observation group (97.56%) (*P* < 0.05).

RETRACTED

**Conclusion:**

The implementation of systematic nursing intervention is conducive to improve the cognitive function, activity of life, and quality of life of senile dementia patients who have a positive effect, and nursing satisfaction is higher.

## 1. Introduction

Senile dementia is a chronic disease with high clinical incidence in the elderly population [1]. With the development of the society, the aging of the global population is gradually increasing. Many elderly people are suffering from the symptoms of senile dementia, which seriously affects their daily life. According to statistics, healthcare measures for senile dementia patients are insufficient, and even in developed countries, less than 50% of senile dementia patients are diagnosed and treated. It is estimated that by 2040, 80 million people worldwide will have senile dementia [2].

Senile dementia is also a progressive neurodegenerative syndrome, which is characterized by cognitive impairment and decreased cognitive function, which leads to degeneration and apoptosis of nerve cells in the brain and nervous system [3]. Its clinical manifestations include memory impairment, aphasia, impaired visual-spatial skills, executive function impairment, and personality and behavior disorders. Neurodegenerative disease of Alzheimer's patients are usually related to the increase of mortality in the elderly [1, 2].

The pathogenesis of senile dementia is the deposition of amyloid protein, senile plaques, and nerve fiber tangles, leading to degeneration and necrosis of neurons. This kind of injury mainly targets the hippocampus related to memory and cognition, which leads to cognitive dysfunction, including memory, language, and attention [4, 5]. The main pathological changes of Alzheimer's disease are brain degeneration and brain atrophy. With the development of the disease, the self-care ability and cognitive function of the patients in their daily life can decline gradually. It will not only affect the prognosis of patients but also seriously affect the quality of life of patients. Therefore, senile dementia has become a research hotspot in the field of central nervous system injury.

Combined with relevant clinical research and analysis, it is found that efficient and high-quality nursing can improve the quality of life of senile dementia patients, improve their disease, and mediate their degree of disease, which is of great significance for improving and optimizing the treatment of senile dementia. This study compares and analyzes the effects of systematic nursing intervention on the living ability and quality of life of senile dementia patients, which are reported as follows.

RETRACTED

## 2. Materials and Methods

### 2.1. Patients

Using the random number table method, 82 senile dementia patients admitted to our hospital from January 2018 to January 2020 were divided into two groups for nursing intervention analysis. In the control group, 41 patients received routine nursing care. In the observation group, 41 patients received systematic nursing intervention. There was no statistically significant difference in the comparison of general information such as age and sex of all patients, indicating that they were comparable (*P* < 0.05), as given in Table 1. In this nursing experiment, all the patients and their families knew the nursing mode and signed the informed consent.

### 2.2. Treatments

The control group was given routine nursing methods to create a good nursing atmosphere, provide correct medication guidance, and improve patients' lifestyle. Changes in vital signs of patients were observed and recorded, and patients were reported in time if there were abnormalities.

The observation group carried out systematic nursing intervention research and in terms of routine nursing, combined with individual differences, strengthened the nursing extension in the following aspects: first of all, psychological nursing intervention should be done well. The mood of elderly patients changes greatly, and they are easily influenced by the external environment. Among them, anxiety and depression are the main mental disorders affecting the daily activities and quality of life of elderly patients with senile dementia [6, 7], nurses' psychological nursing intervention for patients. First, by observing the patient “sitting, walking, and small movements,” determine the patient' anxiety or depression, and with the help of music, activities, and psychological guidance, give the patients more care and encourage patients to communicate with people around them, so that they feel safe, respected, and dignified [8]. Second, safety nursing, the memory, attention, and cognitive ability of the elderly patients will be seriously decreased, and it is also easy to have bad emotions [9]. Therefore, it is suggested to protect the patients from burns or self-injury. It is suggested that the nursing staff should install antiskid escalators in the toilet and the entrance of the corridor and ensure the floor is clean to prevent patients from falling [10]. It is required that the patient's family members or nurses should strengthen the supervision of the patient's medication and prevent the phenomenon of accidental taking of drugs. For patients with severe dementia, it is suggested to take feeding measures, control their diet, and give them more digestible food to prevent incomplete accidents from happening. Third, in nursing life, the nursing staff should ensure that the ward is clean and the noise is low. Because the patient's self-care ability is poor, it is suggested to leave more clothes for patients, encourage patients to change clothes and wash his face, and gradually improve the patient's self-care ability. Adjust the diet reasonably to meet the nutritional intake, strengthen exercise, strengthen body resistance, and promote the metabolism. Finally, health education and nursing should be carried out, and patients and their families should be actively taught disease-related knowledge and nursing methods, so as to promote the effective treatment for patients and reduce the risk of bad behavior and mental health outcomes [11].

RETRACTED

### 2.3. Evaluation Indicators

The Montreal Cognitive Assessment Scale (MoCA) was used to assess the patients' cognition in eight aspects including visual-spatial executive function, naming, memory, attention, language, abstract ability, and directional ability. The total score was 30 points. The higher the score was, the better the cognitive function would be. Barthel index refers to the measurement of the functional status of the patient's daily activities, and the individual score depends on a series of independent behaviors [12]. Barthel index is a commonly used ADL evaluation method in American rehabilitation institutions. The higher the score, the better the functional status of the patients' daily activities. SF-36 is a universal measurement scale developed by the medical outcomes study. Comparing the SF-36 of the two groups, the higher the score, the higher the quality of life [13]. Symptom Checklist-90-Revised (SCL-90-R) was used to assess mental distress [14]. SCL-90-R is one of the most famous mental health test scales in the world. It is currently the most widely used outpatient mental health test scale for mental disorders and mental illness. It can be used to know the degree of mental health in 10 aspects. Social-Adaptive Functioning Evaluation (SAFE) and Social Skills Checklist (SSC) were used to evaluate the social interaction ability of patients before and after nursing intervention. The higher the total score of SAFE indicates the lower the social adaptability of the patients, and the higher the total score of SSC indicates the lower the social skills of the patients. Nursing satisfaction was distributed to patients in the form of a self-prepared nursing satisfaction questionnaire for scoring. The nursing satisfaction after intervention in two groups was evaluated with four grades: very satisfied (above 80 points), basic satisfied (60–80 points), general (40–59 points), and poor (below 40 points). Total satisfaction = (very satisfied + basic satisfied + general)/total cases × 100%. The flow of experiment is shown in Figure 1.

RETRACTED

### 2.4. Statistics Methods

Results were obtained using SPSS 22.0 (SPSS Co., Ltd., Chicago, USA) for statistical analysis. Count data were expressed by (rate), and the chi-square test was used for their comparison between groups. Measurement data were expressed as (mean ± standard deviation), and the *t*-test was used for pairwise comparison, and one-way analysis of variance was used for intergroup comparison. Repeat measures were used for intergroup comparison at the same time point. *P* value less than 0.05 was considered statistically significant.

## 3. Results

### 3.1. Comparison of MoCA Scores before and after Nursing Intervention

After the nursing intervention, the MoCA scores of patients in the two groups were higher than those before the nursing intervention, and the scores in the observation group were higher than those in the control group, and the differences were statistically significant (*P* < 0.05), as shown in Figure 2.

### 3.2. Comparison of Functional Status of Life Activities before and after Nursing Intervention

After the nursing intervention, the Barthel index scores of patients in both groups were higher than that before the nursing intervention, and the observation group was higher than the control group, with statistically significant differences (*P* < 0.05), as shown in Figure 3.

### 3.3. Comparison of Quality of Life before and after Nursing Intervention

After nursing intervention, SF-36 scores of patients in both groups were higher than those before nursing intervention, and those in the observation group were higher than those in the control group, with statistically significant differences (*P* < 0.05), as given in Table 2.

### 3.4. Comparison of Mental Health before and after Nursing Intervention

After nursing intervention, the SCL-90-R scores of patients in both groups were lower than those before nursing intervention, and those in the observation group were lower than those in the control group, with statistically significant differences (*P* < 0.05), as given in Table 3.

### 3.5. Comparison of Outcomes of Social Adaptation before and after Nursing Intervention

After the nursing intervention, the SAFE scores of the two groups were lower than those before the nursing intervention, and the observation group was lower than the control group, with statistically significant differences (*P* < 0.05), as shown in Figure 4.

RETRACTED

### 3.6. Comparison of Scores of Social Skills before and after Nursing Intervention

After nursing intervention, the SSC scores of patients in the two groups were all lower than those before nursing intervention, and the observation group was lower than the control group, with statistically significant differences (*P* < 0.05), as shown in Figure 5.

### 3.7. Comparison of Nursing Satisfaction Scores after Nursing Intervention

After nursing intervention, the total satisfaction of the control group (80.49%) was lower than that of the observation group (97.56%), and the difference was statistically significant (*P* < 0.05), as given in Table 4.

## 4. Discussion

In recent years, with the aging of the population in China, the incidence of senile dementia has increased year by year. By 2050, the elderly population is expected to include 152 million people with dementia [15]. Senile dementia is a group of primary degenerative brain diseases of unknown etiology. The prevalence of these diseases increases with age in the elderly [16]. The onset of senile dementia is slow, difficult, and irreversible, which mainly affects the intelligence and memory of patients, leading to memory loss, and seriously affects the cognition and emotion of patients. Most of the patients with senile dementia will have changes in their behavior and cognitive function within a certain period of time. At present, there is no clear conclusion on its pathogenesis in clinical research, which is mostly due to the influence of people's irregular diet, high pressure of life, and other factors. Good nursing intervention is beneficial to improve the prognosis of patients, alleviate the deterioration of the condition, and significantly enhance the therapeutic effect. In this study, a systematic nursing intervention model was implemented for senile dementia patients to explore the positive effects on the quality of life and living ability of patients.

With the development of dementia, the ability to control one's own life is becoming weaker and weaker, and the quality of nursing influences or determines the quality of life decisively. Conventional health education intervention is too simple in the form of education. Patients are often not impressed by the precautions, dosage, and usage of oral education, resulting in an unsatisfactory nursing effect [17]. Quality of care supports quality of life. Systematic nursing models can be patient-centered, through the evaluation of their condition and disease awareness, combining with individual differences to develop personalized, targeted nursing interventions, strengthen safety education, reduce the occurrence of accidents, and improve nursing safety. The purpose of this nursing is to pay attention to the personality of dementia patients and enable them to live independently and participate in social and cultural activities for as long as possible. Care for people with dementia should be guided by their personal experiences while adapting to their current situation and residual capacity [18].

RETRACTED

MoCA is an evaluation tool used for rapid screening of cognitive dysfunction [19]. The results showed that the MoCA scores of patients in the two groups after nursing intervention were higher than those before nursing intervention. The MoCA score of the systematic nursing intervention observation group was higher than that of the conventional nursing intervention control group. Practice has proved that the systematic nursing intervention had a more positive effect on patients' psychological state and cognitive function, and through continuous training, patients' cognitive ability has been improved.

Under the situation that the general trend of memory decline is hard to be reversed, active, systematic, and effective rehabilitation training can slow the development speed of memory decline. Preventing dementia patients from interrupting rehabilitation training during hospitalization after discharge will affect the therapeutic effects. Therefore, patients with senile dementia need continuous and systematic care to improve their quality of life [20, 21]. After nursing intervention, the Barthel index score and SF-36 score of the two groups were higher than those before nursing intervention, proving that simple nursing could improve the activities of daily living of patients with senile dementia. In addition, in this study, the increases of the Barthel index score and SF-36 score in the observation group were greater than those in the control group, proving that systematic nursing intervention was more conducive to the recovery of patients' daily activities and functional states and was more positive for the improvement of patients' quality of life than conventional nursing intervention.

SCL-90-R is a fully verified and widely used psychological evaluation method [19]. In our study, after nursing intervention, the scores of SCL-90-R in both groups were lower than before nursing intervention, proving that simple nursing can improve the mental health of patients with senile dementia. In addition, in our research, the SCL-90-R scores in the observation group decreased more than those in the control group, especially in depression and anxiety. The average score of the control group was still in mild symptoms, while the average score of the observation group was in a completely negative result. It is proved that systematic nursing intervention is more beneficial to patients' psychological recovery than routine nursing intervention. After nursing intervention, the SAFE scores of both groups were lower than that before the nursing intervention, which proved that the patients with senile dementia needed nursing, because simple nursing can improve the patients' social adaptability. In addition, in this study, the decrease amplitude of the SAFE score and SSC score in the observation group was greater than that in the control group, proving that systematic nursing intervention was more positive for improving the social skills and social adaptability of patients. At the same time, we conducted a nursing satisfaction survey on the patients and found that the total satisfaction of the control group (80.49%) was lower than the total satisfaction of the observation group (97.56%), which proved that the patients were more satisfied with the systematic nursing intervention. It is possible that the systematic nursing intervention is people-oriented and provides more personalized nursing.

RETRACTED

## 5. Conclusion

In our study, MoCA, Barthel index, SF-36, SCL-90-R, SAFE, SSC, and nursing satisfaction were used to evaluate systematic nursing intervention. After discussion, we found that the implementation of systemic nursing interventions in the clinical treatment of senile dementia patients is conducive to improving the patient's intellectual status, cognitive function, daily life activity function, quality of life, psychological status, social adaptability, and social skills, and at this time, the nursing satisfaction is higher. It is proved that systematic nursing intervention has positive influence on cognitive function, life activity ability, and life quality of senile dementia patients and has a promotion value.

## Figures and Tables

**Figure 1:** Experimental flowchart.

**Figure 2:** Comparison of MoCA scores before and after nursing intervention. Compared with before nursing intervention in the same group, ^*∗*^*P* < 0.05. Compared with the control group at the same stage, ^#^*P* < 0.05.

**Figure 3:** Comparison of functional status of life activities before and after nursing intervention. Compared with before nursing intervention in the same group, ^*∗*^*P* < 0.05. Compared with the control group at the same stage, ^#^*P* < 0.05.

**Figure 4:** Comparison of outcomes of social adaptation before and after nursing intervention. Compared with before nursing intervention in the same group, ^*∗*^*P* < 0.05. Compared with the control group at the same stage, ^#^*P* < 0.05.

RETRACTED

**Figure 5:** Comparison of scores of social skills before and after nursing intervention. Compared with before nursing intervention in the same group, ^*∗*^*P* < 0.05. Compared with the control group at the same stage, ^#^*P* < 0.05.

**Table 1:** Comparison of general data of patients (*n*, mean ± SD).

Group	Gender (male/female)	Age (years)	Course of disease (years)	Education year (years)
Control group (*n* = 41)	22/19	67.34 ± 6.60	8.42 ± 1.63	12.19 ± 3.52
Observation group (*n* = 41)	17/24	69.23 ± 6.28	8.91 ± 1.98	12.57 ± 3.19
*t*/*χ*^*2*^ value	1.222	1.328	1.223	0.512
*P* value	0.269	0.188	0.225	0.610

**Table 2:** Comparison of quality of life before and after nursing intervention (*n*, mean ± SD).

SF-36 scores	Control group (*n* = 41)		Observation group (*n* = 41)	
	Before nursing intervention	After nursing intervention	Before nursing intervention	After nursing intervention
Physical functioning	61.24 ± 6.05	68.23 ± 6.54^*∗*^	59.12 ± 5.94	80.23 ± 7.95^*∗*#^
Role-physical	57.09 ± 5.67	70.16 ± 7.09^*∗*^	58.22 ± 5.98	79.45 ± 7.26^*∗*#^
Bodily pain	55.30 ± 5.04	65.18 ± 6.54^*∗*^	56.03 ± 5.22	71.35 ± 7.38^*∗*#^
General health	60.65 ± 6.01	70.65 ± 7.04^*∗*^	60.90 ± 6.30	78.96 ± 7.44^*∗*#^
Vitality	61.06 ± 6.09	70.54 ± 7.08^*∗*^	60.26 ± 6.11	80.57 ± 8.43^*∗*#^
Social functioning	65.46 ± 6.44	71.34 ± 7.20^*∗*^	64.89 ± 6.35	78.96 ± 7.01^*∗*#^
Role-emotional	44.97 ± 4.21	51.96 ± 5.34^*∗*^	45.23 ± 4.35	71.46 ± 7.54^*∗*#^
Mental health	66.25 ± 6.26	71.98 ± 7.23^*∗*^	66.98 ± 6.54	79.23 ± 8.07^*∗*#^
Reported health transition	35.42 ± 3.49	48.75 ± 4.59^*∗*^	33.96 ± 3.28	68.77 ± 7.03^*∗*#^

Notes: compared with before nursing intervention in the same group, ^*∗*^*P* < 0.05. Compared with the control group at the same stage, ^#^*P* < 0.05.

**Table 3:** Comparison of mental health before and after nursing intervention (*n*, mean ± SD).

SCL-90-R scores	Control group (*n* = 41)		Observation group (*n* = 41)	
	Before nursing intervention	After nursing intervention	Before nursing intervention	After nursing intervention
Somatization	1.95 ± 0.16	1.57 ± 0.17^*∗*^	1.89 ± 0.13	1.23 ± 0.14^*∗*#^
Obsessive-compulsive	1.56 ± 0.13	1.23 ± 0.12^*∗*^	1.50 ± 0.15	1.05 ± 0.16^*∗*#^
Interpersonal sensitivity	2.44 ± 0.31	1.68 ± 0.14^*∗*^	2.49 ± 0.16	1.39 ± 0.17^*∗*#^
Depression	2.94 ± 0.35	2.03 ± 0.21^*∗*^	2.92 ± 0.34	1.73 ± 0.23^*∗*#^
Anxiety	2.86 ± 0.33	2.16 ± 0.22^*∗*^	2.96 ± 0.29	1.66 ± 0.16^*∗*#^
Hostility	1.97 ± 0.20	1.66 ± 0.15^*∗*^	1.91 ± 0.24	1.27 ± 0.12^*∗*#^
Phobic anxiety	2.01 ± 0.23	1.83 ± 0.17^*∗*^	2.09 ± 0.21	1.46 ± 0.16^*∗*#^
Paranoid ideation	1.94 ± 0.18	1.64 ± 0.19^*∗*^	1.89 ± 0.17	1.24 ± 0.11^*∗*#^
Psychoticism	1.65 ± 0.12	1.26 ± 0.11^*∗*^	1.61 ± 0.16	1.08 ± 0.15^*∗*#^

Notes: compared with before nursing intervention in the same group, ^*∗*^*P* < 0.05. Compared with the control group at the same stage, ^#^*P* < 0.05.

RETRACTED

**Table 4:** Comparison of nursing satisfaction scores after nursing intervention (*n*, %).

Groups	Nursing satisfaction scores					*χ* ^*2*^	*P*
	Very satisfied	Basic satisfied	General	Poor	Total satisfaction		
Control group (*n* = 41)	9	10	14	8	33 (80.49)	4.493	0.034
Observation group (*n* = 41)	20	12	8	1	40 (97.56)		

## Data Availability

The data used to support the findings of this study are available from the corresponding author upon request.
